# Flash Therapy for Cancer: A Potentially New Radiotherapy Methodology

This article has been retracted.

**DOI:** 10.7759/cureus.46928

**Published:** 2023-10-12

**Authors:** Georgiy Georgievich Polevoy, Devika S Kumar, Sushma Daripelli, Muthu Prasanna

**Affiliations:** 1 Department of Physical Education, Moscow Polytechnic University, Moscow, RUS; 2 Department of Research and Development, Saveetha Institute of Medical and Technical Sciences (SIMATS), Chennai, IND; 3 Department of Anatomy, Government Medical College (GMC) Jangaon, Jangaon, IND; 4 Department of Pharmaceutical Biotechnology, Surya Group of Institutions, Tamil Nadu, IND

**Keywords:** reactive-oxygen-species, flash effect, ultra-high-dose-rate, flash, flash radiotherapy

## Abstract

In traditional treatment modalities and standard clinical practices, FLASH radiotherapy (FL-RT) administers radiation therapy at an exceptionally high dosage rate. When compared to standard dose rate radiation therapy, numerous preclinical investigations have demonstrated that FL-RT provides similar benefits in conserving normal tissue while maintaining equal antitumor efficacy, a phenomenon possible due to the 'FLASH effect' (FE) of FL-RT. The methodologies involve proton radiotherapy, intensity-modulated radiation treatment, and managing high-throughput damage by radiation to solid tissues. Recent results from animal studies indicate that FL-RT can reduce radiation-induced tissue damage, significantly enhancing anticancer potency. Focusing on the potential benefits of FL proton beam treatment in the years to come, this review details the FL-RT research that has been done so far and the existing theories illuminating the FL effects. This subject remains of interest, with many issues still needing to be answered. We offer a brief review to emphasize a few of the key efforts and difficulties in moving FL radiation research forward. The existing research state of FL-RT, its affecting variables, and its different specific impacts are presented in this current review. Key topics discussed include the biochemical mechanism during FL therapy, beam sources for FL therapy, the FL effect on immunity, clinical and preclinical studies on the protective effect of FL therapy, and parameters for effective FL therapy.

## Introduction and background

The majority of patients, with approximately 50% of all malignant cases, receive radiation using X-rays (photons). Ionizing radiation used in radiation treatment destroys cancer cells by inflicting damage on both healthy and malignant cells. Local solid tumors, such as those found in neck and head cancer, skin cancer, lymphoma, lung cancer, and esophageal cancer, are most commonly treated with this form of radiotherapy. Additionally, radiotherapy can serve as an adjuvant therapy, complementing chemotherapy and surgery in treating various conditions, including gastrointestinal tumors, breast cancer, and cervical cancer [1]. Radiation-induced toxicity restricts the tumor's dose, thereby limiting the ability of radiotherapy to suppress tumor development. Furthermore, radiotherapy's prolonged toxicity critically impairs patients' mental and physical health [2]. Nevertheless, the main drawback of RT is that while it is intended to deliver a lethal dose to cancerous cells, exposure to those radiations can damage healthy tissues and cause serious health problems in the short and long term. Conventional radiotherapy employs an external radiation beam, which diminishes in dose as it penetrates patient tissue, unfortunately administering a higher dose to the healthy tissue preceding a deep-seated tumor than to the tumor itself. Moreover, if the beam passes through the tumor, the healthy tissue behind and around the tumor may also receive a significant radiation dose. This can be fatal for sensitive tissues and organs. Ultra-high-dose rate (UHDR) radiation therapy, alternatively referred to as FLASH therapy (FT), has been progressively garnering attention as an emerging technique since 2014, aimed at expanding the therapeutic window. FT delivers doses of radiation at extremely high rates (>40 Gy/s), which are much higher than the typical dose rates used in clinical practice (5 Gy/min). FT has been shown to spare healthy tissue by reducing radiation burden while killing tumor cells [3-6]. The "Flash Effect (FE)" is a phenomenon that describes this sparing of healthy tissue during FT, though the precise mechanisms underpinning the FE are not fully understood. Furthermore, it is thought to be due to several factors, including the rapid cell death in tumor cells at high dose rates and the reduced damage to healthy cells caused by the shorter exposure time. FT is still in the early stages of development, but it has shown promising results in several in vivo studies. It is a potential new cancer treatment option that could help reduce radiotherapy's side effects. Several preclinical experiments revealed that tumor control remained unaffected by variations in dose rate. However, normal tissue showed less damage from the radiation of various modalities when the same dosage was applied at ultra-high mean dose rates above 40 Gy/s [7]. For several preclinical animal studies, FLASH (FL) investigations have been carried out employing a variety of modalities and delivery methods [8]. Investigations into the behavior of tumor tissue have spanned various contexts, including orthotopic glioblastoma tumors, pancreatic cancer cells, and neck and head cancer cells [9]. This review primarily envelops key themes, including the FE, mechanism of the FE, effective FL beam source, and parameters for effective FL-RT.

## Review

FLASH effect (FE)

When dosage is administered using FT at extremely high dose rates as compared to the typical dose rates used in clinical practice, the FE reduces the tissue toxicities precipitated by radiation. According to Normal Tissue Sparing, the FT preserved the neurogenic milieu in an early study. It supported neurogenesis in the normal mice, whereas mice exposed to standard dose rate radiation showed significantly lower levels of undeveloped and mature neural cells within four months after exposure [10]. Additionally, it was claimed that considering the deficiency of final-stage necrosis at nine months of treatment, the dose modulation factor for FL was >1.36 versus conventional dose rates, with comparable outcomes being attained for both 34 Gy FL and 25 Gy at unadventurous dose rates [11]. Tumor control may suggest that more doses might be given to radio-resistant cancers because of FL radiotherapy's higher therapeutic index. Further research is needed for larger patient studies associating FL with traditional dose rate irradiation and research into the best and optimal radiation source and machinery for treating malignancies. Oxygen depletion radiation or hypoxic radiosensitization radiation is delivered at a high dose rate, making the oxygen to be depleted in cancer cells. This depletion creates a hypoxic environment, making cancer cells more radiation-sensitive [12]. DNA damage cells have mechanisms to repair DNA damage caused by radiation. However, when radiation is delivered at a high dose rate, cells do not have time to repair the damage, causing death [13]. When radiation is delivered at a high dose rate, it can delay cell proliferation in the cell cycle process, making them more susceptible to cell death. Various cell death pathways, such as apoptosis and autophagy, can be triggered by radiation, leading to the apoptosis of cancer cells. The rapid radiation dosing not only inhibits cells from repairing DNA damage but also creates a hypoxic condition in tumor tissue, increasing the cancer cells' sensitivity to radiation [14]. The FE may also involve the activation of protective mechanisms in normal cells.

Mechanism of FE

Despite the precise biochemical processes that cause the FE, which are still not fully understood, the emerging paradigm suggests that oxygen plays a crucial role in the biological reaction to FL irradiation. In general, indirect DNA damage from ionizing radiation happens when water undergoes radiolysis, producing reactive oxygen species (ROS) such as hydroxyl radicals that target DNA [15]. According to an early reported study, 30-40% of DNA impairment instigated by low linear-energy-transfer (LET) radiation, such as photons and electrons, is caused by the radiation directly interacting with DNA, whereas 60-70% is instigated by the production of ROS [16]. This secondary DNA destruction is brought on by an interaction with a free radical (such as the hydroxyl radical); the damage is repaired by the survival of molecular oxygen mediated by the production of even more harmful peroxyl radicals [17]. In reality, this is a vital factor of how hypoxic tumors exhibit higher radio-resistance than well-oxygenated tumors, which exhibit an oxygen amplification ratio of 2:3. It has been previously proposed that in the biology of Reactive Oxygen Species (ROS) and free radicals, two additional oxygen-related products differ between normal tissue and malignancies, contributing to the FE (FE). An early study, which exposed zebrafish embryos to either FL (one pulse of 1.8 X 10-6 s) or standard dosage rate (0.1 Gy/s) electron irradiation, demonstrated that FL exerted a smaller impact on the zebrafish's morphology five days post-fertilization, attributable to diminished ROS formation [18]. Moreover, recent studies have spotlighted disparities in redox chemistry and free radical generation to clarify the disparate biological responses of normal and malignant tissue to FL. Furthermore, immunological and inflammatory responses are fundamental processes that significantly contribute to the impact of the FL. A key pro-inflammatory cytokine called transforming growth factor-beta (TGF-β) was specifically linked to changing the impacts of FL compared to traditional dose-rate radiation [19]. TGF-signaling was previously reported to be reduced in mice exposed to FR compared to animals exposed to standard dose rates. The specific effects of conventional radiation on the antitumor immune response remain up for discussion. However, it is known that TGF-β and the accompanying signaling pathway play a critical part in this process. Therefore, for the therapeutic use of FL, especially when radiotherapy is paired with immunotherapy, the changes seen in TGF signaling and immune system activation following FL irradiation require a more thorough investigation. FL‑RT mechanisms are related to oxygen, and their related mechanisms are discussed in Figure 1.

**Figure 1:** Illustration of ROS and the oxygen consumption. Hypothesis of high-dose transitory radiation decreases oxygen levels, and this impact is more pronounced in normal cells, strengthening their radiation resistance; In this hypoxic environment, normal cells experience a decrease in ROS levels, leading to damage to DNA, RNA, proteins, and lipids, while concurrently experiencing an increase in protective NROS levels, which mitigate DNA damage. ROS: Reactive Oxygen Species; NROS: Non-reactive Oxygen Species. Image Credits: Muthu Prasanna Sr. (Corresponding Author).

Effective FL beam source

The FE has mostly been shown in low-energy electron linacs (linear accelerators). Platforms for experimental and medical electron accelerator research are easily accessible. The Kinetron and the Oriatron eRT6 are two specialized electron systems that produce pulsed beams of 4-5 MeV and 4.9-6 MeV electrons, respectively [20]. Using external beam electron FL-RT, deep-seated malignancies can be treated by increasing the electron beam's energy to very-high-energy electrons (VHEE) in the hundreds of MeV range. Recent ultra-high dose rate (UHDR) proton beam innovations have primarily involved hospital-based proton radiation systems, apart from the development in one research center using low-energy proton beams [21]. These therapeutic systems offer high proton energies exceeding 200 MeV, enabling them to cure deep-seated cancers. Therefore, the FL-sparing effects might be advantageous to the normal tissue in the beam path. A revolutionary new technology called the Pluridirectional High-energy Agile Scanning Electron Radiotherapy (PHASER) boasts a compact, power-efficient linear accelerator and radio-frequency (RF) power sources with beam outputs that are hundreds of times greater than those of traditional medical linear accelerators [22]. These novel accelerator devices may eventually be developed with quick RF power distribution systems that send beams in several directions. Delivering treatments in a very conformal manner is possible with ion beam radiation. Upon assessment of proton beams, heavy ion beams feature a sharper lateral penumbra and Bragg peak. An FL beam emits radiation with a high dose rate exceeding 40 Gy/s and features a brief exposure duration [23]. Radiation treatment has been identified to be more effective when utilizing FL beams, thus instigating further research in the field of radiobiology. Produced using an electron linear accelerator, these beams are employed across numerous cell-based biomedical studies. The entire beam illumination dosage during tests must be monitored in real-time. The charge density created in the device's cavity is too high to monitor FL beams when using a normal transmission-type monitor chamber because the electrometer overflows [24]. The mean pulse intensity per unit chamber volume and unit dosage for 6-MeV FL electron beams with a pulse duration of 2.5 s is calculated to be approximately 14 mA/(cm3Gy) [25]. Conventional electrometers cannot accommodate such substantial input currents. In this study, a system capable of measuring pulse current for monitoring 6-MeV FL electron beams was constructed using a PTW-7862 ionization chamber. The system comprises a digital voltmeter, a high-input-resistance buffer amplifier, a current-integrating capacitor, and a polarization voltage generator. Measurements employing the prototype device were conducted on 6-MeV FL electron beams, generating voltage signals correlating to the number of pulses. Future signal processing studies are requisite to enhance the practical application of the device.

FE on immunity

Lymphopenia usually results from high-dose clinical radiation. The most radiosensitive cell types among adult hematopoietic cell populations are lymphocytes, such as T, B, and NK cells. When human peripheral blood mononuclear cells are exposed ex vivo to 2 Gy of radiation, approximately 50% of the T cells undergo apoptosis 24 hours post-exposure [26]. The number of CD3 T cells in individuals' peripheral blood mononuclear cells was considerably reduced after receiving a total body dose of 12 Gy of radiation. In contrast, CD14 monocyte numbers largely remain unaffected, underscoring the pronounced radio-sensitivity of circulating lymphocytes [27]. The blood volume inside the irradiated zone determines the proportion of destroyed immune cells when irradiation time is less than blood circulation time. The proportion of destroyed immune cells is calculated using a combination of the blood volume within the irradiated organs and the blood volume that flows into the irradiated organs, applicable when the irradiation period exceeds the blood circulation time. The FL-sparing effect on circulating immune cells amplifies in a dose-dependent manner, with a projected sparing impact following a single dose of 5, 10, 20, and 30 Gy. It is noteworthy that the blood circulation time contravenes the minimal dosage rate necessary to produce the FE [28]. Due to longer blood circulation times in humans compared to mice, the authors hypothesized that the lowest dosage rate to protect circulating immune cells would be lower in humans [29]. Creating immune-stimulatory medicines or agents blocks immune suppressor components and respective pathways. Both groups of medications are coupled with radiation to expand the potential application of radiotherapy beyond its conventional usage to provide local control or cure. Anti-PDL1, anti-CTLA4, anti-OX40, and combination blocking with several agents are immune-modifying medication classes used in conjunction with radiation [30].

Parameters for effective FL-RT

In order to produce the FE, radiation dosage rates that are several orders of magnitude greater than usual must be used. Several other considerations must also be taken into account. These variables encompass the total dosage given, pulse rate, length, width, number, and total delivery time. The radiation's source, utilized in numerous contemporary FL experiments employing electron linear accelerators, is another crucial factor. A long-term function for the FL impact, particularly on chronic inflammation, has been suggested by the observation that the rising dosage rate decreased the amount of prematurely senescent cells (measured by -galactosidase positive cells) and reduced the stimulation of TGF- expression [31]. Subsequently, it was shown that the variation in proton dosage rate did not impact immediate biological outcomes, such as clonogenic survival and the development of H2AX foci [32]. Although the result was not statistically significant, there was an indication of reduced clonogenic survival at both FL dosage rates compared to the conventional dose rate. Modifications in endpoints, such as cell cycle progression, chromosomal abnormalities, ROS levels, DNA damage signaling, and DNA damage foci associated with the production of DSBs following FL, may be crucial to understanding the underlying processes that generate the FE. The specialized equipment of FL-RT requires equipment that can deliver ultra-high radiation dose rates. Additional research is necessary to fully comprehend the FE and confirm its safety and efficacy in humans. The need to develop new treatment planning techniques, such as conventional radiation therapy treatment planning techniques, may be different for FL-RT. New techniques must be developed to ensure the radiation is delivered safely and effectively to the tumor.

Clinical and preclinical studies

In recent studies, the antitumor efficiency of FL-RT gave many promising results that are summarized below.

Brain

In a study by Montay-Gruel P et al. (2020), FL-RT had a similar antitumor effect to conventional RT in mice with glioblastoma but with a protective effect on cognitive function [33]. In another study by Montay-Gruel P et al. (2019), FL-RT was found to have no effect on cognitive function in mice without tumors [34]. In a study by Simmons DA et al. (2019), FL-RT was found to have a protective effect on cognitive function in mice with glioblastoma. This result emphasizes the therapeutic equivalence and competence of FL-RT, suggesting that it can effectively target and destroy tumor cells within the brain, just like the traditional radiation therapy approach. FL-RT, in comparison to conventional delivery time irradiation, exhibited a reduction in cognitive impairment and the associated neurodegeneration. This effect may be attributed to a lower level of neuroinflammation induction, indicating a hopeful strategy for enhancing the therapeutic effectiveness in treating brain tumors with radiation therapy.

Intestine

In a study by Venkatesulu BP et al. (2019), FL-RT did not have a protective effect on toxicity or survival in mice with intestinal cancer [35]. In a study by Loo BW et al. (2017), among the 101 mice exposed to radiation doses ranging from 13 to 19 Gy, the survival rate for conventional radiation treatment was 29% (49 mice) compared to an impressive 90% survival rate after FL-RT (59 mice) [36]. Those studies highlight that FL-RT was tested as a potential treatment option in mice with intestinal cancer. The results of these experiments indicated that FL-RT not only appeared to be safe, with minimal harm to healthy tissues, but also established clinical effectiveness in treating intestinal cancer. This finding could be a significant step in developing FL-RT as a therapeutic approach for human patients with intestinal cancer. However, further research and clinical trials would be needed to confirm its safety and efficacy in humans.

Lung

In a study by Fouillade C et al., FL-RT was found to have a protective effect on normal lung tissue in mice with lung cancer [37]. In a study by Favaudon V et al., FL-RT was found to have a similar antitumor effect to conventional RT in mice with lung cancer but with a protective effect on normal lung tissue [3]. Normal lung tissues refer to the healthy, non-cancerous cells and structures within the lung. Human lung fibroblast is a type of cell found in the connective tissue of the lungs [38]. They play a role in maintaining the structural integrity of the lung tissue. When these cells are exposed to radiation, they can be damaged, leading to potential complications or adverse effects. So, when the statement mentions that FL-RT has a protective effect on normal lung tissue in human lung fibroblasts, it suggests that when they are exposed to FL-RT, they experience less damage or harm compared to traditional radiotherapy techniques, which is a significant finding because it implies that FL-RT may offer a safer and more tissue-sparing option for treating lung cancers or other lung-related conditions, as it helps to protect healthy lung tissue while still targeting cancerous cells. Further research and clinical trials would be necessary to fully validate these findings and assess the potential clinical applications of FL-RT in lung cancer treatment.

Skin

In a study by Bourhis J et al., FL-RT effectively treated a patient's lymphoma [39]. In a study by Vozenin MC et al. in the year 2018, FL-RT was found to be effective in treating squamous carcinoma in a cat [5]. The successful treatment of a patient indicates that FL-RT has the potential for clinical use in treating lymphoma. It may open doors to further research, clinical trials, and the incorporation of FL-RT into standard cancer treatment protocols [40]. It is important to note that while this is promising, clinical findings need to be supported and corroborated by additional studies and research, including large-scale clinical trials, to establish FL-RT as a standard and widely accepted treatment option for lymphoma and other types of cancer. Nonetheless, this finding represents a positive step forward in developing innovative and potentially more effective therapies for cancer patients.

Blood

In a study by Chabi S et al., FL-RT was found to have a similar antitumor effect to conventional RT in mice with leukemia but with a protective effect on normal hematopoiesis [41]. The protective effect on normal hematopoiesis is particularly important because one of the challenges in treating leukemia is mitigating adverse effects and damage to healthy blood-forming cells [42]. FL-RT's ability to protect these cells may lead to fewer side effects and complications for individuals. Hematopoiesis is the process by which the body forms new blood cells, including RBCs, WBCs, and platelets. Thus, it suggests that FL-RT had a protective effect on this normal blood cell formation process. In other words, while effectively treating leukemia, FL-RT appeared to spare or protect the healthy blood-forming cells in the bone marrow.

Other Cancers

In a preclinical study by Bubley G et al., FL-RT effectively killed prostate cancer cells [43]. In a study by Beyreuther E et al., FL-RT was found to be safe and effective in zebrafish embryos [44]. Overall, the results of these studies suggest that FL-RT is a promising new treatment modality with the potential to improve the therapeutic index of RT. However, further research is needed to confirm these findings and to optimize the use of FL-RT in clinical practice. Despite numerous extensive preclinical animal studies regarding FL, the limitations of FL in human investigations remain prominently apparent (Figure 2).

**Figure 2:** Investigations involving animals treated with FL and restrictions on human research. Research in mice, cats, and zebrafish has encouraged the advancement of FL radiation. There are still a number of challenges in exploring utilization its application in humans, including considerations related to dosage, equipment, radiation source, and financial aspects. Image Credits: Muthu Prasanna Sr. (Corresponding Author).

## Conclusions

Rapid oxygen depletion induced by FL-RT leads to momentary hypoxia. However, the distinct responses between healthy and malignant tissues remain unclear. FL-RT may reduce radiation dosages to healthy tissue, and innovative and promising strategies for combining radiotherapy with other anticancer therapies may be encouraged. More animal studies are required before FL-RT can become the primary radiation technique utilized in clinical settings. The transition should be altered to accommodate larger radiotherapy fields, conformal radiation across multiple fields, redefinition of safe dose limits for healthy tissue, and radical cancer dosage irradiation. More studies are necessary for FL-RT to be applied to medical practice to benefit cancer patients, especially at physiological oxygen concentrations.
